The article "Alterations in CD8+ Tregs, CD56+ Natural Killer Cells and IL-10 Are Associated With Invasiveness of Nonfunctioning Pituitary Adenomas (NFPAs)" was published in 2021. Journal: Pathol Oncol Res.

# Alterations in CD8^+^ Tregs, CD56^+^ Natural Killer Cells and IL-10 Are Associated With Invasiveness of Nonfunctioning Pituitary Adenomas (NFPAs)

**DOI:** 10.3389/pore.2021.598887

**Published:** 2021-03-25

**Authors:** Xinmei Huang, Jiong Xu, Yueyue Wu, Li Sheng, Yue Li, Bingbing Zha, Tiange Sun, Ju Yang, Shufei Zang, Jun Liu

**Affiliations:** ^1^ Department of Endocrinology, The Fifth People’s Hospital of Shanghai, Fudan University, Shanghai, China; ^2^ Department of Pathology, The Fifth People’s Hospital of Shanghai, Fudan University, Shanghai, China

**Keywords:** invasive nonfunctioning pituitary adenomas, immune tolerance, CD8 + tregs, natural killer cells, IL-10

## Abstract

Invasive nonfunctioning pituitary adenomas (NFPAs) grow rapidly and the mechanisms are unclear. Among many complex mechanisms, the role of immunity in the development of NFPAs has not been fully explored. Here, we analyzed the clinical features 146 NFPA patients who underwent trans-sphenoidal surgery or craniotomy and examined the effects of immune tolerance in invasiveness of NFPA patients using fluorescence-activated cell sorting and immunohistochemical methods. We found patients with invasive NFPAs had more visual deficits and defective fields, higher tumor size, and lower white blood cell count compared with patients with noninvasive NFPAs. Additionally, compared with patients with noninvasive NFPAs, patients with invasive NFPAs had conspicuously lower CD3^−^CD56^+^ natural killer (NK) cells and significantly higher levels of CD3^+^CD8^+^CD28-T cells (CD8^+^ Tregs) and interleukin-10 (IL-10) in peripheral blood. Moreover, patients with invasive NFPAs had lower infiltrated CD56^+^ cells, less infiltrated CD28^+^ cells, and significantly greater IL-10 expression. These results demonstrated that low CD56^+^ cells infiltration and CD28^+^ cells infiltration, as well as high IL-10 expression in pituitary tumor tissues, were related with increased invasiveness of NFPAs. Levels of CD3^−^CD56^+^ NK cells, CD8^+^ Tregs and IL-10 in the peripheral blood could be feasible diagnostic markers for invasive NFPAs.

## Introduction

Pituitary adenomas (PAs) account for 10–25% of all intracranial neoplasms [1]. They are derived from intracranial adenohypophyseal cells and often presented as neurological deficits (particularly visual impairment), pituitary dysfunction, parasellar compartment invasion and sphenoid sinuses [2]. Although the majority of PAs are histologically benign, 25–55% of PAs often invade surrounding structures and exhibit malignant behaviors [3, 4]. Up to now, neurosurgery resection remains the initial treatment of choice for most PAs. However, curative radical surgery of invasive PAs remains difficult. Furthermore, approximately 10–20% PAs are unable to produce active hormone and classified as nonfunctioning pituitary adenomas (NFPAs) [5]. As hormone inactivity leads to delayed diagnosis, the incidence of invasive NFPAs becomes higher. In addition, the efficiency of NFPAs chemotherapy is unsatisfactory and there is no consensus regarding the radiotherapy. Therefore, it is urgent to elucidate the mechanisms of the biological behavior of PAs, especially for NFPAs, thereby developing an effective treatment for them [6].

Immune tolerance or escape is pivotal in tumor development, progression, and control [7, 8] and mediated by both deletion of self-reactive T cells and activation of suppressing T-cell activity [9]. Studies of brain tumor-infiltrating lymphocytes (TILs) have provided evidence demonstrating that the immune system is naturally involved in the immune surveillance of brain tumors [10–12]. Pituitary adenomas are the second most common type of intracranial tumor. Recently, pituitary adenomas have been found [13–16] to have varying degrees of immune cell infiltrates. Greater infiltration of CD68^+^ macrophages could increase the production of CD4^+^ regulatory T cells (Tregs) to suppress the immune system [17, 18] and is associated with increased invasiveness of adenomas [16]. The study have demonstrated that down-regulation of transforming growth factor-beta (TGFβ, one of the main immune suppressive mediators) is correlated with tumorigenesis process of NFPAs [19]. However, the role of immunity in the development of NFPAs has not been fully explored. Accordingly, in this study, we examined the clinical characteristics of patients with NFPAs and assessed the effects of inflammatory or immune cells on invasive NFPAs.

## Methods

### Participants and Samples

A total of 146 patients with NFPAs who underwent transsphenoidal surgery or craniotomy and 20 healthy controls at the Fifth People’s Hospital of Shanghai, Fudan University between 2012 and 2016 were included in this study. Age and sex-matched 20 normal subjects were selected from physical examination center of our hospital. Patients who had undergone previous drug therapy or radiation therapy or had a recurrence or pituitary apoplexy were excluded. Patients were also excluded if they were taking medications that could influence immune function, such as glucocorticoids and immunosuppressants. Patients with obesity, diabetes mellitus, severe hypertension, infectious diseases, severe hepatic and renal dysfunctions and other malignant tumors were also excluded. The diagnosis of NFPAs was based on clinical symptoms and signs including amenorrhea, oligomenorrhea, galactorrhea, infertility, hirsutism, acne, enlargement of the hands and feet, headaches, and vision loss as well as hormonal levels, magnetic resonance imaging, histopathological examination, and immunohistochemical staining for all anterior pituitary hormones. To evaluate changes in the percentages of lymphocytes and levels of cytokines, 2 ml of ethylenediaminetetraacetic acid-anticoagulated whole blood and 4 ml of procoagulant serum were collected from the 146 patients with NFPAs and 20 healthy controls. The surgical adenomas specimens were also obtained from the 146 patients with NFPAs to assess the infiltration of lymphocytes, and expression of inflammatory cytokines in adenomas. The study protocol was approved by the Ethics Committee of Shanghai Fifth People’s Hospital, Fudan University (2014029), and all participants gave written informed consent to participate in the study in accordance with the Declaration of Helsinki.

### Pituitary Imaging, Hormone Analysis, and Cytokine Testing

MRI was used to measure the diameters of NFPAs and evaluate tumor invasion. Tumor invasiveness was assessed based on Hardy’s classification. Only grade III and IV tumors were considered as invasive NFPAs. Serum levels of follicle-stimulating hormone (FSH), luteinizing hormone (LH), estradiol (E_2_), testosterone (T) and prolactin (PRL) were examined using electrochemiluminescence immunoassays and serum levels of growth hormone (GH), thyroid-stimulating hormone (TSH), free thyroxine (FT_4_), adrenocorticotropin (ACTH), and cortisol (F) were examined using chemiluminescence assays. Serum levels of interferon-γ (IFN-γ), interleukin-2 (IL-2), and interleukin-10 (IL-10) were measured by enzyme-linked immunosorbent assay (ELISA; Raybio) according to the manufacturer’s protocols.

### Lymphocyte Subtype Analysis by Fluorescence Activated Cell Sorting

The T-cell subtypes were determined using FACS analysis. In brief, whole blood samples were lyzed with Lymphoprep™ (STEMCELL Technologies, Vancouver, Canada). Lymphocytes were stained with 100 μL phosphate-buffered saline (PBS) containing 1% bovine serum albumin (BSA) and 0.1% NaN_3_, together with 5 μL PerCPcy5.5-conjugated anti-human CD3 (cat. no.45-0037-42), followed by simultaneous staining with 5 μL fluorescein isothiocyanate (FITC)-conjugated anti-human CD4 (cat. no. 11-0049-42) or APC-conjugated anti-human CD8 (cat. no. 17-0086-42) and phycoerythrin (PE)-conjugated anti-human CD28 (cat. no. 12-0289-42) or FITC-conjugated anti-human CD56 (cat. no. 11-0566-42; all eBioscience). The cells were then incubated for 20 min at 4°C, and flow cytometry was performed using a BD FACS Calibur flow cytometer (BD Biosciences, Franklin Lakes, NJ, United States).

### Immunohistochemistry

The surgical specimens were processed to 5 μm sections using conventional formalin-fixed, paraffin-embedded method. These sections were dewaxed, boiled for 20 min in citrate buffer (10 mM, pH 6.0) to retrieve antigens, and subjected to immunohistochemical staining for CD3 (cat. no. GB13014; antibody dilution 1:50; Servicebio), CD4 (cat. no. GB13064-1; antibody dilution 1:25; Servicebio), CD8 (cat. no. GB13068; antibody dilution 1:50; Servicebio), CD28 (cat. no. ab113358; antibody dilution 1:100; Abcam), CD56 (cat. no. 14255-1-Ap; antibody dilution 1:100; Proteintech), IL-10 (cat. no. GB13108; antibody dilution 1:400; Servicebio), IFN-γ (cat. no. 5365-1-Ap; antibody dilution 1:100; Proteintech), and IL-2 (cat. no. ab92381; antibody dilution 1:250; Abcam) according to the manufacturer’s protocol. In brief, primary antibodies were incubated overnight at 4°C followed by horseradish peroxidase (HRP)-labeled, anti-rabbit antibodies for 50 min (Dako) and visualized using diaminobenzidine tetrachloride (Dako). The sections were then photographed using a computer-assisted video-imaging system (NIKON DP controller, Japan). A total of 20 random fields of each stained specimen were examined to calculate the product of immunoreactivity intensity and the proportion of lymphocytes positive staining, the mean integrated optical density (IOD) value and mean optical density (MOD) of inflammatory cytokines using Image-Pro Plus 6.0 software (Media Cybernetics, Inc., Rockville, MD, United States). The MOD is equal to IOD/Area. The intensity of the immunoreactivity (IR) was stratified into four categories: 0, no IR; 1, canary yellow IR; 2, pale brown IR; and 3, tan IR. The proportion of positive cells was classified into four groups: 0, 0–5% of cells exhibiting IR; 1, 6–25% of cells exhibiting IR; 2, 26–50% of cells exhibiting IR; 3, 51–75% of exhibiting IR; 4, >75% of cells exhibiting IR.

### Statistical Analysis

The data are expressed as the mean ± standard error of mean (SEM) or as number (percent). Continuous variables were compared using One-way analysis of variance (ANOVA) test followed by least significant difference (LSD) and Mann-Whitney U tests. Categorical variables were compared using Chi-square tests. Spearman’s rank correlation was used to evaluate the relationships between continuous variables. Differences with *p* value <0.05 were considered statistically significant. All statistical analyses were performed using SPSS software, version 21 (IBM, Chicago, IL, United States) and Graph Pad Prism 5 software.

## Results

### Demographic and Clinical Characteristics

A total of 146 patients with NFPAs who underwent transsphenoidal surgery or craniotomy and 20 healthy controls were evaluated in the present study. These patients had a mean age of 58 years old, 66 (39.8%) women and 100 (60.2%) men. Of the 146 NFPA patients, 86 (58.9%) had invasive NFPAs, and 60 (41.1%) had noninvasive NFPAs (Table 1). Patients with invasive or noninvasive NFPAs had significantly higher PRL level (24.89 ± 1.77, 19.98 ± 2.35, and 10.24 ± 0.86, respectively), but lower levels of LH (5.52 ± 0.70, 6.67 ± 0.96, and 20.11 ± 4.91, respectively) and FSH (15.24 ± 2.03, 15.13 ± 2.62, and 39.24 ± 9.90, respectively) than healthy controls. Although visual deficits and visual field defects are the most common symptoms in all patients with NFPAs, they were more common in patients with invasive NFPAs than in patients with noninvasive NFPAs. In addition, patients with invasive NFPAs had significantly larger tumor size than patients with noninvasive NFPAs (29.71 ± 0.86 and 17.90 ± 0.69, respectively). Moreover, patients with invasive NFPAs had significantly lower level of white blood cells than patients with noninvasive NFPAs and healthy controls (5.63 ± 0.17, 6.30 ± 0.19, and 6.62 ± 0.17, respectively).

**TABLE 1:** Demographic and clinical characteristics of 146 patients with NFPAs.

	Control (*n* = 20)	Noninvasive NFPAs (*n* = 60)	Invasive NFPAs (*n* = 86)	*p* value
Age	57.75 ± 1.14	57.93 ± 1.86	57.56 ± 1.20	0.983
Sex, no. (%)				0.355
Female, no. (%)	10 (50.0%)	20 (33.3%)	36 (41.9%)	—
Male, no. (%)	10 (50.0%)	40 (66.7%)	50 (58.1%)	—
Symptom, no. (%)				0.006
Headache	—	34 (56.7%)	33 (38.4%)	—
Visual field defect	—	4 (6.7%)	20 (23.3%)	—
Visual deficit	—	27 (45.0%)	62 (72.1%)	—
Nausea and vomiting	—	6 (10.0%)	11 (12.8%)	—
Polyuria	—	4 (6.7%)	1 (1.3%)	—
None		7 (8.1%)	7 (11.7%)	—
SBP (mmHg)	124.70 ± 3.18	126.83 ± 2.00	124.38 ± 1.74	0.639
DBP (mmHg)	73.10 ± 1.57	77.03 ± 1.16	76.86 ± 1.06	0.216
BMI (kg/m^2^)	22.70 ± 0.48	23.83 ± 0.40	23.39 ± 0.31	0.222
Tumor size (mm)	—	17.90 ± 0.69	29.71 ± 0.86^a^	<0.001
WBC (×10^^9^/L)	6.62 ± 0.17	6.30 ± 0.19	5.63 ± 0.17^ab^	0.003
PRL (µg/L)	10.24 ± 0.86	19.98 ± 2.35^c^	24.89 ± 1.77^b^	0.003
GH (µg/L)	0.81 ± 0.23	0.71 ± 0.15	0.59 ± 0.09	0.597
LH (IU/L)	20.11 ± 4.91	6.67 ± 0.96^b^	5.52 ± 0.70^b^	<0.001
FSH (IU/L)	39.24 ± 9.90	15.13 ± 2.62^b^	15.24 ± 2.03^b^	<0.001
E_2_ (pg/ml)	14.17 ± 2.92	22.02 ± 2.22	17.33 ± 1.55	0.094
T (ng/ml)	2.64 ± 0.77	2.16 ± 0.31	1.07 ± 0.15^ab^	0.001
ACTH (pg/ml)	25.61 ± 2.27	26.39 ± 2.26	23.73 ± 1.35	0.527
F (nmol/L)	295.01 ± 19.59	340.59 ± 34.12	312.96 ± 21.77	0.641
TSH (mIU/L)	2.61 ± 0.44	1.53 ± 0.17^b^	1.75 ± 0.15^c^	0.015
FT_4_ (pg/ml)	1.18 ± 0.05	1.42 ± 0.15	1.36 ± 0.11	0.644

Data are presented as mean ± SEM or number (percent). ^a^ *P* < 0.01 *vs*. noninvasive NFPAs, ^b^ *P*<0.01 *vs*. control, ^c^ *P*<0.05 *vs*. control. Continuous variables except tumor size were compared using One-way ANOVA followed by LSD. Tumor size was compared using Mann-Whitney U tests. Categorical variables were compared using Chi-square tests. Abbreviations: ACTH, adrenocorticotropin; BMI, body mass index; DBP, diastolic blood pressure; E_2_, estradiol; F, cortisol; FSH, follicle-stimulating hormone; FT_4_, free thyroxine; LH, luteinizing hormone; GH, growth hormone; NFPAs, nonfunctioning pituitary adenomas; PRL, prolactin; SBP, systolic blood pressure; T, testosterone; TSH, thyroid-stimulating hormone; WBC, while blood cell.

### Determination of CD3^+^CD4^+^ and CD3^+^CD8^+^ T-Cell Subpopulations Using FACS Analysis in NFPAs

In order to detect the immune responses in patients with NFPAs, peripheral T cell subsets including CD3^+^CD4^+^T lymphocytes and CD3^+^CD8^+^T lymphocytes were analyzed using FACS. As shown in Figure 1, the percentage of CD3^+^CD4^+^ T cells were not significantly altered among healthy controls, patients with noninvasive NFPAs, and patients with invasive NFPAs. Patients with invasive NFPAs had higher percentage of CD3^+^CD8^+^ T cells than patients with noninvasive NFPAs and healthy controls, but not significantly. Additionally, neither the percentage of CD3^+^CD4^+^ nor the percentage of CD3^+^CD8^+^ cells was correlated with tumor size (*r* = −0.163, *p* = 0.612 and *r* = 0.253, *p* = 0.428, respectively).

**FIGURE 1:** Distribution and differences of T cell subpopulations among healthy controls (*n* = 20), patients with noninvasive NFPAs (*n* = 60) and patients with invasive NFPAs (*n* = 86). Neither the percentage of CD3^+^CD4^+^ nor the percentage of CD3^+^CD8^+^ cells was not significantly altered among the three groups. Bars represent means ± SEMs. In-NFPAs, invasive nonfunctioning pituitary adenomas; Non-NFPAs, noninvasive nonfunctioning pituitary adenomas.

### CD3^−^CD56^+^ NK Cells Were Decreased and CD3^+^CD8^+^CD28^−^ T Cells Were Increased in Peripheral Blood of Patients With Invasive NFPAs

The percentage of peripheral CD3^−^CD56^+^ NK cells and CD3^+^CD8^+^ CD28^−^ T cells are shown in Figure 2. It is clear from the figures that patients with invasive NFPAs had significantly lower percentage of CD3^−^CD56^+^ NK cells, but higher percentage of CD8^+^ Tregs than patients with noninvasive NFPAs and healthy controls, but patients with noninvasive NFPAs showed no significant differences in CD3^−^CD56^+^ NK cells and CD8^+^ Tregs compared with healthy controls. In addition, neither CD3^−^CD56^+^ NK cells nor CD8^+^ Tregs were correlated with tumor size (*r* = −0.321, *p* = 0.365 and *r* = 0.377, *p* = 0.184, respectively).

**FIGURE 2:** Distribution and differences of CD3^−^CD56^+^ NK cells and CD3^+^CD8^+^CD28^−^ T cells (CD8^+^ Tregs) among healthy controls (*n* = 20), patients with noninvasive NFPAs (*n* = 60) and patients with invasive NFPAs (*n* = 86). Percentage of CD3^−^CD56^+^ NK cells was significantly lower in patients with invasive NFPAs than patients with noninvasive NFPA and healthy controls. Patients with invasive NFPAs had a significantly higher level of CD8^+^ Tregs than patients with noninvasive NFPAs and healthy controls. Bars represent means ± SEMs. **p < 0.01, *p < 0.05. In-NFPAs, invasive nonfunctioning pituitary adenomas; Non-NFPAs, noninvasive nonfunctioning pituitary adenomas.

### Level of IL-10 Was High in Peripheral Blood of Patients With Invasive NFPAs

Th1 cytokines activate macrophages, NK cells, and cellular immunity, whereas Th2 cytokines tend to promote the humoral immune responses. IL-10 is mainly produced by Th2 cells and thought to be an immunosuppressive factor. In the present study, the production of IFN-γ and IL-2 Th1 cytokines, and IL-10 in peripheral blood were examined using ELISA. As shown in Figure 3, patients with invasive NFPAs had significantly higher IL-10 levels than patients with noninvasive NFPAs and healthy controls. However, there were no significant differences in IFN-γ and IL-2. Moreover, none of the IL-10, IFN-γ, or IL-2 level was correlated with tumor size (*r* = 0.024, *p* = 0.925; *r* = −0.115, *p* = 0.568; and *r* = −0.232, *p* = 0.276, respectively).

**FIGURE 3:** Differences in levels of cytokines among healthy controls (*n* = 20), patients with noninvasive NFPAs (*n* = 60) and patients with invasive NFPAs (*n* = 86). Level of IL-10 was significantly higher in patients with invasive NFPAs than in patients with noninvasive NFPAs and healthy in controls. Bars represent means ± SEM. *p < 0.05. LnIFN-γ represents the natural logarithm of IFN-γ, LnIL-2 represents natural logarithm of IL-2, LnIL-10 represents natural logarithm of IL-10. In-NFPAs, invasive nonfunctioning pituitary adenomas; IFNγ, interferon-γ; IL-2, interleukin-2; IL-10, interleukin-10; Non-NFPAs, noninvasive nonfunctioning pituitary adenomas.

### Lower Infiltration of CD56^+^ Cells and CD28^+^ Cells but Greater Expression of IL-10 in Tumor Tissues of Patients With Invasive NFPAs

To further explore the role of immune tolerance or escape in IPAs, infiltration of lymphocytes and expression of inflammatory cytokines in pituitary adenomas specimens were analyzed. As shown in Figure 4B, the infiltration of CD3^+^, CD4^+^, and CD8^+^ cells were similar in patients with invasive NFPAs and noninvasive NFPAs. Moreover, Figure 4B showed that patients with invasive NFPAs exhibited significantly lower infiltration of CD56^+^ cells and CD28^+^ cells than patients with noninvasive NFPAs. IL-10 is an immunosuppressive factor, whereas both IL-2 and IFN-γ are proinflammatory cytokines. Our results showed that patients with invasive NFPAs had significantly higher expression of IL-10, lower expression of IFN-γ and IL-2 than patients with noninvasive NFPAs, but not significantly different [Figure 4B].

**FIGURE 4:** Photomicrograph and expression differences of CD3^+^ cells, CD4^+^ cells, CD8^+^ cells, CD56^+^ cells, CD28^+^ cells and inflammatory cytokines in tumor tissue of NFPAs. Brown indicates positive staining. **(A)** Photomicrograph of CD3^+^, CD4^+^, CD8^+^, CD56^+^, CD28^+^ cells and inflammatory cytokines in tumor tissue of patients with noninvasive NFPAs (*n* = 60) and patients with invasive NFPAs (*n* = 86); **(B)** Expression differences of CD3^+^, CD4^+^, CD8^+^, CD56^+^, CD28^+^ cells and inflammatory cytokines between two groups, indicating lower infiltrated CD56^+^ cells, less infiltrated CD28^+^ cells, and significantly greater IL-10 expression in patients with invasive NFPAs. Bars represent means ± SEMs. **p < 0.01, *p < 0.05. In-NFPAs, invasive nonfunctioning pituitary adenomas; IFNγ, interferon-γ; IL-2, interleukin-2; IL-10, interleukin-10; IOD, integrated optical density; MOD, Mean Optical Density is equal to IOD/Area; Non-NFPAs, noninvasive nonfunctioning pituitary adenomas.

## Discussion

As suggested in the present study, the majority of NFPAs are macroadenomas and come to clinical attention due to mass effects, such as headaches, visual field defect, visual deficit, and hypopituitarism. The invasiveness of pituitary adenomas has been correlated to age, tumor size, sex, and tumor type [6, 20]. However, our results only showed that tumor size was related with invasiveness of NFPAs as a common type of PAs. Moreover, our results also showed that the level of WBC, which contains several important immune cells and play vital roles in immune function, was lower in patients with invasive NFPAs than patients with noninvasive NFPAs, suggesting that tumor immunity could have an important role in invasiveness of NFPAs.

T cell subsets include CD3^+^CD4^+^ T cells and CD3^+^CD8^+^ T cells. CD4^+^ Th cells and CD8^+^ cytotoxic T cells play important roles in inhibiting and impeding tumor growth and killing tumor cells (as shown in Table 2). Some studies have suggested that the presence of CD4^+^ and CD8^+^ cells were correlated with improved survival in patients with certain cancers [10, 21–23]. Effector CD8^+^ cytotoxic T cells have been shown to be specifically associated with favorable prognosis of patients with some malignant tumors, such as glioblastomas, ovarian cancers and pancreatic cancers [22, 24, 25]. Programmed death-ligand 1 (PD-L1), as an immunosuppressive protein, was expressed highly in tumor tissue of PA patients [26], which can induce immune evasion by desensitizing the recognition and elimination of tumor cells via CD8^+^ T cells [27]. In addition, Hazrati et al. [28] reported that Th1 activator adjuvants and autoantigens are successful for treatment of patients with recurrent pituitary macroprolactinoma after operation. Our results showed that there were no statistically significant differences in the percentage of CD3^+^CD8^+^ T cells and the infiltration of CD8^+^ cells between patients with noninvasive NFPAs and patients with invasive NFPAs, suggesting that CD8^+^ cytotoxic T cells were not associated with invasiveness of NFPAs.

**TABLE 2:** Immunological role of several immune cells and inflammatory cytokines.

Parameters	Immunological role
CD3^+^CD4^+^T lymphocytes and CD3^+^CD8^+^T lymphocytes	As the subsets of T cell, CD3^+^CD4^+^T lymphocytes and CD3^+^CD8^+^T lymphocytes play important roles in inhibiting and impeding tumor growth and killing tumor cells. However, neither one of them were associated with invasiveness of NFPAs in our study
CD3^−^CD56^+^ NK cells	As a central component of the innate immune system, CD3^−^CD56^+^ NK cells as a subtype of NK cells control several types of tumors by inhibiting tumor cell dissemination. Our findings indicated that the reduction of NK cells was related with increased invasiveness of NFPAs and may be a useful biomarker of invasive NFPAs
CD8^+^CD28^−^ cells (CD8^+^ tregs)	As a common subset of tregs, CD8^+^ tregs that render antigen presenting cells (APC), mainly dendritic cells (DCs), tolerant through cell-cell contact, can secrete IL-10, TGF-β, IFN-γ, CCL4, and directly kill CD4^+^ effector T cells and APCs. Our findings suggested that high level of CD8^+^ tregs and low infiltration of CD28^+^ cells were associated with the invasiveness of NFPAs. CD8^+^ tregs may be another important biomarker for the invasion of NFPAs
IL-10	IL-10 is mainly produced by Th2 cells. As an immunosuppressive factor that is generally thought to support tumor growth and progression. Similarly to CD8^+^ tregs and CD56^+^ NK cells, high expression of IL-10 in tumor tissue was also related with increased invasiveness of NFPAs. IL-10 may present a useful biomarker for diagnosis of invasive NFPAs
IFN-γ and IL-2	Th1 cells can secrete IFN-γ and IL-2, which activate macrophages, NK cells, and cellular immunity, and play important role in protection against tumor cells. But neither one of them were associated with invasiveness of NFPAs in our study

CCL4, chemokine C-C motif ligand 4; IL-10, interleukin-10; IL-2, interleukin-2; IFN-γ, interferon-γ; TGF-β, transforming growth factor-β; NFPAs, nonfunctioning pituitary adenomas; NK, natural killer.

As a central component of the innate immune system, NK cells control several types of tumors by inhibiting tumor cell dissemination (as shown in Table 2) [29]. However, to our best knowledge, studies of the effects of NK cells on solid tumors are limited [23, 30–33]. Ma et al showed that NK cells are infiltrated in prolactinomas and non-secreting pituitary adenomas [15]. In this study, we assessed the frequencies of peripheral CD3^−^CD56^+^ NK cells as a subtype of NK cells and showed that patients with invasive NFPAs had significantly lower percentage of CD3^−^CD56^+^ NK cells than patients with noninvasive NFPAs and healthy controls, and less tumor infiltration of CD56^+^ cells than patients with noninvasive NFPAs. Although it is unclear whether alterations of NK cells in invasive NFPAs are the cause or responses to the adenoma, these results still indicated that a lower percentage of NK cells and lower infiltration of NK cells were related with increased invasiveness of NFPAs. The levels of CD3^−^CD56^+^ NK cells may be a useful biomarker of invasive NFPAs.

Not all T cells are antitumor effector immune cells. For example, Tregs [34, 35], including natural CD4^+^CD25^+^ Tregs (nTregs), T helper 3 (Th3) cells, type 1 Tregs (Tr1 cells), and CD8^+^CD28^−^ cells (CD8^+^ Tregs), could induce immune tolerance by suppressing host immune responses and thus inhibit effective antitumor immune responses CD8^+^ Tregs (as shown in Table 2) is a common subset of Tregs and induce immune tolerance of antigen presenting cells (APC), primarily dendritic cells (DCs), through cell-cell contact. Additionally, these cells can secrete IL-10 [35], transforming growth factor (TGF)-β, IFN-γ, and chemokine C-C motif ligand 4, and directly kill CD4^+^ effector T cells and APCs. Previous studies [36–38] have shown that patients with non-small cell lung cancer (NSCLC) had higher percentage of CD8^+^ Tregs than healthy controls and that this T-cell subset is correlated with pathological stage of NSCLC. Wu et al [39] have found similar results in ovarian cancer, demonstrating that patients with ovarian cancer had higher percentage of CD8^+^ Tregs than patients with benign ovarian tumors. To the best of our knowledge, our study is the first to demonstrate that patients with invasive NFPAs had significantly higher percentage of peripheral CD8^+^ Tregs than patients with noninvasive NFPAs and healthy controls and lower tumor infiltration of CD28^+^ cells than patients with noninvasive NFPAs. Therefore, our findings exhibited that higher level of CD8^+^ Tregs and lower infiltration of CD28^+^ cells were associated with the invasiveness of NFPAs. Furthermore, CD8^+^ Tregs may be another important biomarker for the invasion of NFPAs, and also promote NFPAs growth and progression by inhibiting the immune response against cancer. Similar to CD56^+^ NK cells, further investigation is needed to prove that alterations of CD8^+^ Tregs in invasive NFPAs may be the cause of invasive NFPAs in the future.

The Th1-type immune response plays important role in protection against tumor cells [10, 21, 23]. Cytokines can reflect the populations of immune effector cells to a certain degree. Th1 cells can secrete IFN-γ and IL-2 (as shown in Table 2), which activate macrophages and are related to the generation of CTLs. In contrast, IL-10 [40] (as shown in Table 2) is an acting immunosuppressive cytokine that is generally thought to support tumor growth and progression. Our results showed that patients with invasive NFPAs had higher IL-10 expression both in peripheral blood and tumor tissue than those with noninvasive NFPAs, which indicates that IL-10 may play a vital role in the development of NFPAs and present a useful biomarker for diagnosis of invasive NFPAs.

## Conclusion

In conclusion, the infiltrations of immune cells and expression of inflammatory cytokine were different between noninvasive NFPAs and invasive NFPAs. Low infiltration of CD56^+^ and CD28^+^ cells, as well as high expression of IL-10 in tumor tissue, were related with increased invasiveness of NFPAs. Moreover, according to the results of lymphocytes and inflammatory cytokine in peripheral blood, our findings also indicated that the levels of peripheral CD3^−^CD56^+^ NK cells, CD8^+^ Tregs and IL-10 may be useful biomarkers for diagnosis of invasive NFPAs.

## Data Availability

All datasets presented in this study are included in the article/Supplementary Material.

## References

[1] Loyo-VarelaMHerrada-PinedaTRevilla-PachecoFManrique-GuzmanS. Pituitary tumor surgery: review of 3004 cases. World Neurosurg (2013) 79 (2), 331–6. 10.1016/j.wneu.2012.06.024 22732515

[2] BronsteinMDMelmedS. Pituitary tumorigenesis. Arq Bras Endocrinol Metabol (2005) 49 (5), 615–25. 10.1590/s0004-27302005000500003 16444345

[3] SyroLVRotondoFRamirezADi IevaASavMARestrepoLM Progress in the diagnosis and classification of pituitary adenomas. Front Endocrinol (Lausanne) (2015) 6, 97. 10.3389/fendo.2015.00097 26124750PMC4464221

[4] ChatzellisEAlexandrakiKIAndroulakisIIKaltsasG. Aggressive pituitary tumors. Neuroendocrinology (2015) 101 (2), 87–104. 10.1159/000371806 25571935

[5] DekkersOMHammerSde KeizerRJRoelfsemaFSchuttePJSmitJW The natural course of non-functioning pituitary macroadenomas. Eur J Endocrinol (2007) 156 (2), 217–24. 10.1530/eje.1.02334 17287411

[6] MelmedS. Pathogenesis of pituitary tumors. Nat Rev Endocrinol (2011) 7 (5), 257–66. 10.1038/nrendo.2011.40 21423242

[7] CharlesNAHollandECGilbertsonRGlassRKettenmannH. The brain tumor microenvironment. Glia (2012) 60 (3), 502–14. 10.1002/glia.21264 22379614

[8] ReimanJMKmieciakMManjiliMHKnutsonKL. Tumor immunoediting and immunosculpting pathways to cancer progression. Semin Cancer Biol (2007) 17 (4), 275–87. 10.1016/j.semcancer.2007.06.009 17662614PMC2742305

[9] SinghNJSchwartzRH. Primer: mechanisms of immunologic tolerance. Nat Clin Pract Rheumatol (2006) 2 (1), 44–52. 10.1038/ncprheum0049 16932651

[10] DunnGPDunnIFCurryWT. Focus on TILs: prognostic significance of tumor infiltrating lymphocytes in human glioma. Cancer Immun (2007) 7, 12. 17691714PMC2935751

[11] LampsonLA. Brain tumor immunotherapy: an immunologist's perspective. J Neurooncol (2003) 64 (1-2), 3–11. 10.1007/BF02700015 12952281

[12] JacobsJFIdemaAJBolKFNierkensSGrauerOMWesselingP Regulatory T cells and the PD-L1/PD-1 pathway mediate immune suppression in malignant human brain tumors. Neuro-oncology (2009) 11 (4), 394–402. 10.1215/15228517-2008-104 19028999PMC2743219

[13] HeshmatiHMKujasMCasanovaSWollanPCRacadotJVan EffenterreR Prevalence of lymphocytic infiltrate in 1400 pituitary adenomas. Endocr J (1998) 45 (3), 357–61. 10.1507/endocrj.45.357 9790270

[14] RossiMLJonesNREsiriMMHavasLal IzziMCoakhamHB. Mononuclear cell infiltrate and HLA-Dr expression in 28 pituitary adenomas. Tumori (1990) 76 (6), 543–7. 10.1177/030089169007600605 2284689

[15] MaLLiGSuYHeQZhangCZhangJ. The soluble major histocompatibility complex class I-related chain A protein reduced NKG2D expression on natural killer and T cells from patients with prolactinoma and non-secreting pituitary adenoma. J Clin Neurosci (2010) 17 (2), 241–7. 10.1016/j.jocn.2009.05.023 20045334

[16] LuJQAdamBJackASLamABroadRWChikCL. Immune cell infiltrates in pituitary adenomas: more macrophages in larger adenomas and more T cells in growth hormone adenomas. Endocr Pathol (2015) 26 (3), 263–72. 10.1007/s12022-015-9383-6 26187094

[17] WeiJGabrusiewiczKHeimbergerA. The controversial role of microglia in malignant gliomas. Clin Dev Immunol (2013) 2013, 285246. 10.1155/2013/285246 23983766PMC3741958

[18] ZamarronBFChenW. Dual roles of immune cells and their factors in cancer development and progression. Int J Biol Sci. (2011) 7 (5), 651–8. 10.7150/ijbs.7.651 21647333PMC3107473

[19] ButzHLikóICzirjákSIgazPKorbonitsMRáczK MicroRNA profile indicates downregulation of the TGFβ pathway in sporadic non-functioning pituitary adenomas. Pituitary (2011) 14 (2), 112–24. 10.1007/s11102-010-0268-x 21063788

[20] MeijBPLopesMBEllegalaDBAldenTDLawsERJr. The long-term significance of microscopic dural invasion in 354 patients with pituitary adenomas treated with transsphenoidal surgery. J Neurosurg (2002) 96 (2), 195–208. 10.3171/jns.2002.96.2.0195 11838791

[21] ErreniMMantovaniAAllavenaP. Tumor-associated macrophages (TAM) and inflammation in colorectal cancer. Cancer Microenviron (2011) 4 (2), 141–54. 10.1007/s12307-010-0052-5 21909876PMC3170420

[22] SatoEOlsonSHAhnJBundyBNishikawaHQianF Intraepithelial CD8^+^ tumor-infiltrating lymphocytes and a high CD8^+^/regulatory T cell ratio are associated with favorable prognosis in ovarian cancer. Proc Natl Acad Sci USA (2005) 102 (51), 18538–43. 10.1073/pnas.0509182102 16344461PMC1311741

[23] MeleroIRouzautAMotzGTCoukosG. T-cell and NK-cell infiltration into solid tumors: a key limiting factor for efficacious cancer immunotherapy. Cancer Discov (2014) 4 (5), 522–6. 10.1158/2159-8290.CD-13-0985 24795012PMC4142435

[24] LohrJRatliffTHuppertzAGeYDictusCAhmadiR Effector T-cell infiltration positively impacts survival of glioblastoma patients and is impaired by tumor-derived TGF-β. Clin Cancer Res. (2011) 17 (13), 4296–308. 10.1158/1078-0432.CCR-10-2557 21478334

[25] OrhanAVogelsangRPAndersenMBMadsenMTHölmichERRaskovH The prognostic value of tumour-infiltrating lymphocytes in pancreatic cancer: a systematic review and meta-analysis. Eur J Cancer (2020) 132, 71–84. 10.1016/j.ejca.2020.03.013 32334338

[26] WangPWangTYangYYuCLiuNYanC. Detection of programmed death ligand 1 protein and CD8+ lymphocyte infiltration in plurihormonal pituitary adenomas. Medicine (2017) 96 (49), e9056. 10.1097/MD.0000000000009056 29245312PMC5728927

[27] AlsaabHOSauSAlzhraniRTatipartiKBhiseKKashawSK PD-1 and PD-L1 checkpoint signaling inhibition for cancer immunotherapy: mechanism, combinations, and clinical outcome. Front Pharmacol (2017) 8, 561. 10.3389/fphar.2017.00561 28878676PMC5572324

[28] HazratiSMAghazadehJMohtaramiFAbouzariMRashidiA. Immunotherapy of prolactinoma with a T helper 1 activator adjuvant and autoantigens: a case report. Neuroimmunomodulation (2006) 13 (4), 205–8. 10.1159/000100405 17337912

[29] VivierETomaselloEBaratinMWalzerTUgoliniS. Functions of natural killer cells. Nat Immunol (2008) 9 (5), 503–10. 10.1038/ni1582 18425107

[30] HalamaNBraunMKahlertCSpilleAQuackCRahbariN Natural killer cells are scarce in colorectal carcinoma tissue despite high levels of chemokines and cytokines. Clin Cancer Res (2011) 17 (4), 678–89. 10.1158/1078-0432.CCR-10-2173 21325295

[31] CantoniCHuergo-ZapicoLParodiMPedrazziMMingariMCMorettaA NK cells, tumor cell transition, and tumor progression in solid malignancies: new hints for NK-based immunotherapy? J Immunol Res (2016) 2016, 4684268. 10.1155/2016/4684268 27294158PMC4880686

[32] LevyEMRobertiMPMordohJ. Natural killer cells in human cancer: from biological functions to clinical applications. J Biomed Biotechnol (2011) 2011, 676198. 10.1155/2011/676198 21541191PMC3085499

[33] WennerbergEKremerVChildsRLundqvistA. CXCL10-induced migration of adoptively transferred human natural killer cells toward solid tumors causes regression of tumor growth *in vivo* . Cancer Immunol Immunother (2015) 64 (2), 225–35. 10.1007/s00262-014-1629-5 25344904PMC11028951

[34] WangHYWangRF. Regulatory T cells and cancer. Curr Opin Immunol (2007) 19 (2), 217–23. 10.1016/j.coi.2007.02.004 17306521

[35] RodiMDimisianosNde LasticALSakellarakiPDeraosGMatsoukasJ Regulatory cell populations in relapsing-remitting multiple sclerosis (RRMS) patients: effect of disease activity and treatment regimens. Int J Mol Sci (2016) 17 (9). 10.3390/ijms17091398 PMC503767827571060

[36] ChenCChenDZhangYChenZZhuWZhangB Changes of CD4^+^CD25^+^FOXP3^+^ and CD8^+^CD28^−^ regulatory T cells in non-small cell lung cancer patients undergoing surgery. Int Immunopharmacol (2014) 18 (2), 255–61. 10.1016/j.intimp.2013.12.004 24345703

[37] KaragözBBilgiOGümüsMErikçiAASayanOTürkenO CD8^+^CD28^−^ cells and CD4^+^CD25^+^ regulatory T cells in the peripheral blood of advanced stage lung cancer patients. Med Oncol (2010) 27 (1), 29–33. 10.1007/s12032-008-9165-9 19148592

[38] ChenCChenZChenDZhangBWangZLeH. Suppressive effects of gemcitabine plus cisplatin chemotherapy on regulatory T cells in nonsmall-cell lung cancer. J Int Med Res (2015) 43 (2), 180–7. 10.1177/0300060514561504 25659373

[39] WuMChenXLouJZhangSZhangXHuangL Changes in regulatory T cells in patients with ovarian cancer undergoing surgery: preliminary results. Int Immunopharmacol (2017) 47, 244–50. 10.1016/j.intimp.2017.04.004 28437737

[40] TanikawaTWilkeCMKryczekIChenGYKaoJNúñezG Interleukin-10 ablation promotes tumor development, growth, and metastasis. Cancer Res (2012) 72 (2), 420–9. 10.1158/0008-5472.CAN-10-4627 22123924PMC3261323

